The article "How to Perfuse: Concepts of Cerebral Protection during Arch Replacement" was retracted in 2016. Reasons: plagiarized text; overlap with other authors' work.

# How to Perfuse: Concepts of Cerebral Protection during Arch Replacement

**DOI:** 10.1155/2015/981813

**Published:** 2015-12-02

**Authors:** Andreas Habertheuer, Dominik Wiedemann, Alfred Kocher, Guenther Laufer, Prashanth Vallabhajosyula

**Affiliations:** ^1^Division of Cardiovascular Surgery, University of Pennsylvania Medical Center, Philadelphia, PA 19104, USA; ^2^Department of Cardiac Surgery, Vienna General Hospital, Medical University of Vienna, 1090 Vienna, Austria

## Abstract

Arch surgery remains undoubtedly among the most technically and strategically challenging endeavors in cardiovascular surgery. Surgical interventions of thoracic aneurysms involving the aortic arch require complete circulatory arrest in deep hypothermia (DHCA) or elaborate cerebral perfusion strategies with varying degrees of hypothermia to achieve satisfactory protection of the brain from ischemic insults, that is, unilateral/bilateral antegrade cerebral perfusion (ACP) and retrograde cerebral perfusion (RCP). Despite sophisticated and increasingly individualized surgical approaches for complex aortic pathologies, there remains a lack of consensus regarding the optimal method of cerebral protection and circulatory management during the time of arch exclusion. Many recent studies argue in favor of ACP with various degrees of hypothermic arrest during arch reconstruction and its advantages have been widely demonstrated. In fact ACP with more moderate degrees of hypothermia represents a paradigm shift in the cardiac surgery community and is widely adopted as an emergent strategy; however, many centers continue to report good results using other perfusion strategies. Amidst this important discussion we review currently available surgical strategies of cerebral protection management and compare the results of recent European multicenter and single-center data.

## 1. Introduction

It is the delicate anatomic site of the aortic arch, vascular crossroad between body and brain, that intrigues cardiac surgeons as much as demanding both the finest technical skills and thorough knowledge in neurophysiology to deal with pathologies requiring surgical repair. Surgery for complex aortic pathologies, that is, acute dissections and aneurysms extending into the arch, remains one of the technically most challenging endeavors of modern cardiac surgery [1]. Arch reconstruction in the setting of acute type A dissection has historically been associated with significant morbidity, especially in terms of neurologic dysfunction, and mortality due to ischemic end organ damage occurring during the circulatory arrest period; however there is an appreciable recent trend towards improvement. The International Registry for Acute Aortic Dissections (IRAD) reported an in-hospital mortality rate of 26% in 2009 [2] with urgency status and recent history of central neurologic events being important preoperative risk factors and determinants of mortality and neurologic outcome [3, 4]. Only recently the same registry reported an in-hospital mortality rate of 19.7% for acute aortic dissections cumulating the results of 4,428 patients and 28 IRAD centers [5].

Although postoperative results are important in all aspects of cardiovascular surgery, neurologic and mortality outcomes are especially significant in surgery of the thoracic aorta, as these can reflect the circulation management applied as well as the patient's aortic pathology [6]. Reports from several studies have shown that most permanent postoperative neurologic dysfunctions (defined as persistent focal or global neurologic dysfunction with correlating structural abnormalities upon cerebral computed tomography or magnetic resonance imaging) are actually caused by embolic phenomena rather than the cerebral protective regimen applied. Alternatively, transient neurologic dysfunction (defined as the occurrence of postoperative, timely limited confusion, transient motor weakness, seizure, or agitation without correlation with imaging studies and with complete reversal at the time of hospital discharge) has been more closely related to cerebral ischemic times [6–13].

The introduction of profound hypothermia in the mid-1970s by Griepp et al. allowing short periods of complete circulatory arrest paved the way for modern arch surgery requiring prolonged ischemic tolerance of the CNS for extensive aortic repair extending into the transverse arch [14]. Over the past 2 decades various adjunctive techniques of cerebral circulatory management have evolved to increase the safety and duration of cerebral protection. These adjunctive techniques all comprise distinct elaborate selective perfusion protocols (unilateral or bilateral selective ACP and selective RCP, resp.) in combination with various degrees of hypothermic circulatory arrest. The techniques of cerebral protection during surgery of the aortic arch can be divided into those aimed at suppressing the CNS metabolic demand and those aimed at maintaining the metabolic supply during the time of exclusion of the cerebral vessels. More specifically, current protocols include DHCA alone [15, 16], selective RCP [7, 8, 12, 13, 17, 18], and selective ACP [19]. More recently, some centers advocated for the use of more liberal circulatory arrest temperatures and championed the merits of moderate hypothermic circulatory arrest (MHCA) in combination with selective ACP [11, 20–23]. A range of adverse postoperative neurologic outcomes and early mortality is reported for each of these techniques. Postoperative permanent neurologic dysfunction is reported as 4.8% to 12.5% for DHCA [6, 9, 15], 2.4% to 7.1% for selective RCP/DHCA [6, 12, 17, 24, 25], 3.3% to 9.6% for selective ACP/DHCA [6, 9, 11, 12, 19, 23, 26], and 3.2% to 9.6% for selective ACP/modified MHCA [21, 23, 27]. Postoperative mortality is reported as 6.3% to 13.3% for DHCA [9, 15], 2.9% to 10.1% for selective RCP/DHCA [12, 17, 24, 25], 2.0% to 12.7% for selective ACP/DHCA [9, 11, 12, 19, 23, 26], and 9.4% to 11.5% for selective ACP/MHCA [3, 21, 23, 27].

This paper reviews current state-of-the-art neuroprotective strategies and compares elaborate clinical regimens focusing on the benefits of hypothermia and cold antegrade cerebral perfusion. Recent trends in combining ACP with steadily increasing mild-to-moderate hypothermic arrest are discussed from various perspectives and under the light of recent large-cohort trials and multicenter international meta-analyses. The influence of the anticipated time of circulatory arrest on the cerebral protection strategy is discussed as widely adopted by the cardiac surgery community. Predictors of adverse outcomes and determinants of transient neurological dysfunction and permanent neurological dysfunction, respectively, are discussed to leave the reader with a thorough understanding of the current literature as well as current clinical practices.

## 2. Cerebral Protection: A Contemporary Review of Available Surgical Strategies

There is no doubt that adequate cerebral protection during aortic arch exclusion plays a key role in achieving successful outcomes. However, it was a long road of trial and error for cardiac surgery to develop both effective surgical techniques to deal with pathologies of the thoracic aorta and effective cerebral protection regimens. With the first introduction of cardiopulmonary bypass and extracorporal circulation, surgery of the aortic arch seemed to be an impossible undertaking. During the 1950s, De Bakey, Crawford, and Cooley in Houston introduced surgical techniques specifically addressing pathologies of the thoracic and thoracoabdominal aorta, including the transverse arch, and they were the first to report on 6 cases of aortic dissection addressed surgically [28]. However, those techniques did not gain widespread acceptance by that time due to their high technical complexity and limited postoperative outcomes in terms of mortality and neurology. It took another decade for Borst and colleagues [29] to adopt the use of profound hypothermia as an adjunct to cardiopulmonary bypass for closure of an arteriovenous fistula and for Griepp et al. [14] to report on their first routine arch procedures, in profound hypothermia.

### 2.1. Hypothermic Circulatory Arrest

Since the discovery that hypothermia induces neuroprotective effects, it has become a widely adopted concept in cardiovascular surgery in general and in surgery of the thoracic aorta specifically. Systemic hypothermia reduces metabolic tissue rate thereby increasing neuronal ischemic tolerance. Cerebral metabolism is progressively depressed by approximately 6-7% per 1°C decline in core body temperature [1]. The brain's electrical activity starts to decrease at mildly reduced temperatures (<33.5°C) and ceases with profound hypothermia at 19.0°C to 20.0°C with no electrical activity detectable upon assessment on electroencephalogram. Accordingly, the core body temperature is a significant determinant of cerebral metabolic demand and oxygen consumption and, when compared to normothermia, can be reduced anywhere in between >50% at 28°C (moderate hypothermia) and >80% at 18°C (profound hypothermia), respectively [4]. Thus, hypothermia alone prolongs the CNS tolerance to ischemic insults during periods of circulatory arrest. For some time it was tempting to assume that deep hypothermia is sufficient to prevent any neurologic complication; however, this concept had to undergo some major revisions [37]. Results from both experimental and clinical studies suggest that cerebral metabolic suppression and thus neurologic protection during profound hypothermia is less complete than previously suspected [30, 38, 39]. Particularly in the elderly and in patients with preexisting neurologic dysfunctions, DHCA at intervals >25 min was associated with TND, fine motor deficits, and prolonged hospital stays [1, 10]. More recently, Fischer et al. [40] reported that already after 30 min of HCA at 15°C the oxygen saturation of the frontal cortex as measured on near infrared spectroscopy (NIRS) drops below the relatively safe threshold of 60%, increasing the risk of serious adverse outcomes (*p* = 0.038). Neurologic complications occur more frequently following prolonged DHCA of >40 min and may be transient or permanent [1, 10, 41].

In an attempt to calculate the safe durations of circulatory arrest, McCullough et al. [30] used the cerebral metabolic rate by oxygen consumption (CMRO_2_) as an estimate and achieved comparable results of 31 min at 15°C. According to this equation intervals could be extended to 45 min at 10°C (Table 1):

(1) $$\begin{array}{c} {\text{CMRO}}_{2}=\frac{\text{CBF }\times \text{ cerebral AV oxygen difference}}{100} \end{array}$$

In terms of prolonged hypothermic arrest, immediate postoperative coagulation disorders have been reported in literature [42, 43]; however, there remains a lack of scientific proof for this claim [44] and coagulopathy is much rather thought to be triggered by prolonged bypass and extracorporal circulation times than pure hypothermia. In their 2-center comparative study of moderate versus deep HCA in 776 patients, Milewski et al. [6] found no significant difference in the incidence of reoperation for bleeding (profound versus deep HCA: 3.8 versus 4.3%; *p* = 0.783). Similarly, Harrington et al. [44] did not find an increased risk of postoperative bleeding following DHCA.

### 2.2. Selective Cerebral Perfusion, ACP

In 1956, the Houston group successfully used normothermic ACP to resect a large aneurysm of the ascending thoracic aorta via the common carotid arteries [45]. One year later De Bakey et al. [46] reported on the first successful open arch surgery in an attempt to remove a mycotic aneurysm involving both the ascending aorta and the transverse arch using normothermic cerebral perfusion via direct cannulation of both carotid arteries and distal perfusion via cannulation of the right femoral artery. However, this approach of bicarotid perfusion in normothermia was soon to be abandoned due to a high incidence of thromboembolism and consecutive adverse neurological outcome. Following the introduction of routine surgery under profound hypothermia and circulatory arrest in 1975 by Griepp et al. [14], it took another 10 years for Guilmet et al. in Europe and Kazui in Japan to raise aneurysm surgery to the next level: the principle of antegrade cerebral perfusion in combination with hypothermic circulatory arrest resulted in a significantly reduced incidence of neurological complications [47, 48]. The new neuroprotective strategy of “cold cerebroplegia” combined profound (6–12°C) selective cerebral perfusion via the carotid arteries during circulatory arrest in deep hypothermia (26°C) increasing ischemic tolerance and allowing for longer operative times while avowing profound hypothermic body core temperatures. Simultaneously, the Stanford group published their experience with selective ACP and low-flow cerebroperfusion (30 mL/kg/min) at 26–28°C [49]. They used 3 distinct cannulation/perfusion strategies: unilateral via a 14-F cannula directly into the innominate artery with occlusion of both left carotid and left subclavian artery, unilateral via the left carotid, and bilateral via innominate and carotid artery simultaneously.

When considering ACP, further variables need reflection to achieve optimal cerebral protection, that is, target cerebral blood flow (CBF), blood pressure, hemodilution, and intracranial pressure (ICP). At rest, 15% of the cardiac output is estimated to constitute normal cerebral blood flow [50]. Experimental studies highlight the association of increased ICP and consecutive requirements for higher perfusion pressures with cerebral injury and adverse neurological outcome [51] and high cerebral pump blood flows on HCA with high ICPs and cerebral edema alleviating any protective effect [52]. Thus the pump flows and pressures during selective ACP must be adequately balanced. More recently, Jonsson et al. [53] reported on their experimental results of safe minimal CBF during selective ACP and identified an ischemic threshold of at least 6 mL/kg/min. Therefore, most centers adopting ACP into their routine surgical practice perfuse the brain at a rate of approximately 8–12 mL/kg/min and a perfusion pressure of 40–60 mmHg at temperatures between 23 and 28°C [36, 37, 44, 50]. When considering optimal cerebral blood flow another crucial variable is that autoregulation maintains both cerebral blood flow and pressure in a physiologic spectrum under normal circumstances but the organisms' ability to do so is temperature dependent and is dramatically decreased at 25°C and below [1].

### 2.3. Selective Cerebral Perfusion: RCP

Retrograde cerebral perfusion might be used as an adjunct to hypothermic circulatory arrest, yet the use of RCP is source of much wider debate in the cardiac surgery community. The use of RCP was originally reported by Mills and Ochsner [54] for the management of massive arterial air embolism during cardiopulmonary bypass in 1980. In 1990 Ueda et al. [55] first described the routine use of continuous RCP in thoracic aortic surgery for the purpose of cerebral protection during periods of circulatory arrest. Retrograde perfusion is instituted by means of both bicaval cannulation and arterial cannulation, respectively. Arterial cannulation can be achieved directly via the distal ascending aorta, the left axillary artery, or femoral artery, depending on both the patient anatomy and extent of repair. In contrast to ACP, a shunt-line between arterial and venous cannula is employed, which remains clamped during the cooling period. When satisfactory hypothermia is achieved (depending on the institution's guidelines), the arterial line is clamped to engage into circulatory arrest, the superior vena cava (SVC) is snared, and the shunt-line is opened to achieve venous cerebral perfusion, in a retrograde fashion. RCP is usually adjusted to 100–500 mL/min to maintain a central venous pressure of 15–25 mmHg [56]. Desaturated blood from the arch vessels is returned to the heart lung bypass via a cardiotomy sucker.

There is evidence that RCP may accomplish neuroprotection by providing cerebral metabolic support, retrogradely expelling atheromatous and gaseous emboli from the cerebral vasculature and maintaining cerebral hypothermia [57]. However, there remains the concern that very little of the perfusate actually reaches the cerebral microvasculature to provide adequate neuroprotection. In experimental studies led by Ehrlich et al. [58] from the Mount Sinai Medical Center in New York, retrograde cerebral perfusion provided negligible flow through brain capillaries in pigs. Calculations based on the number of fluorescent microspheres trapped in the brain showed flows as low as 0.02 ± 0.02 mL/min/100 g brain parenchyma. Less than 13% of retrograde superior vena caval inflow blood returned to the aortic arch.

## 3. Cerebral Protection: A Strategic Comparison of Current Clinical Practice

Best evidence papers are shown in Table 2. Based on the above reasoning, cerebral protection during arch exclusion may potentially be achieved using various surgical techniques and neuroprotective principles. The therapeutic armamentarium ranges from DHCA, via ACP with moderate to deep hypothermic circulatory arrest, which might be extended from unilateral to bilateral cerebral perfusion (Figure 1) to RCP with deep hypothermic arrest. Recent data from European surveys suggest that moderate hypothermia in combination with selective ACP as opposed to deep hypothermic arrest is an emergent strategy and in fact is the strategy more often used [31, 59].

### 3.1. Antegrade versus Retrograde with DHCA: Does It Matter?

Based on conflicting anatomical, clinical [20], and experimental animal data [58] the effectiveness of RCP to perfuse the brain to an extent as to support aerobic metabolism is still questioned.

Misfeld et al. [36] from the Leipzig Heart Center recently reported on their 6-year, 636-patient experience. They found statistically significant differences in their circulatory arrest times dependent on the perfusion strategy applied: 22 ± 17 minutes for unilateral ACP, 23 ± 21 minutes bilateral ACP, 18 ± 12 minutes for RCP, and 15 ± 13 minutes DHCA (*p* < 0.001). The use of any form of ACP (versus DHCP alone or RCP) was identified as protective against the development of PND by multivariate analysis (odds ratio: 0.4; 95% CI: 0.2 to 0.7; *p* = 0.005) despite longer circulatory arrest times. Early mortality for the entire cohort was 11% (*n* = 72) and was not statistically different between patients receiving different modes of cerebral protection (*p* = 0.2). Multivariate analysis identified acute type A aortic dissection (OR: 2.4; 95% CI: 1.4 to 4.2; *p* = 0.001), history of preoperative myocardial infarction (OR: 2.4; 95% CI: 1.07 to 5.4; *p* = 0.03), total aortic arch replacement with elephant trunk (OR: 1.9; 95% CI: 1.07 to 3.5; *p* = 0.03), and duration of CPB (OR: 1.011 per minute of CPB; 95% CI: 1.007 to 1.01; *p* = 0.01) as independent predictors of early mortality.

Milewski et al. [6] from the Hospital of the University of Pennsylvania, Philadelphia, found slightly contradicting results in terms of PND when comparing their 2-center, 776-patient experience. They found no significant difference in permanent neurologic deficit, temporary neurologic dysfunction, or renal failure, between RCP/DHCA and ACP/MHCA. Mean cerebral ischemic time and visceral ischemic time differed between RCP/DHCA and ACP/MHCA (*p* < 0.001). Increasing arch reconstruction times were associated with a worse neurologic outcome irrespective of the technique applied. For arch reconstructive times less than 45 minutes, univariate analysis revealed no significant difference in permanent neurologic deficit between RCP/DHCA (2.8%) and ACP/MHCA (3.2%). Similar results could be shown for TND.

Ganapathi et al. [60] from the Duke University Medical Center retrospectively compared their 440-patient cohort experience. An unadjusted comparison of the primary endpoints did not reveal any differences in neurologic complications (10.8% ACP versus 7.5% RCP; *p* = 0.36), 30-day in-hospital mortality (3.6% ACP versus 2.5% RCP; *p* = 0.61), or composite 30-day in-hospital major morbidity (17.5% ACP versus 15.0% RCP; *p* = 0.59).

In total, those studies [6, 36, 60] comprised 1852 patients with unequivocal results regarding primary neurological endpoints.

### 3.2. Unilateral versus Bilateral Cerebral Perfusion

Antegrade cerebral perfusion became the method of choice for cerebral protection during aortic arch surgery in many centers in the past decade [9, 26, 61, 62]. Controversies exist with regard to unilateral versus bilateral ACP. This question becomes increasingly imminent when considering pathologies like carotid artery stenosis, previous stroke, or anatomical variants like incomplete circle of Willis with missing anterior of posterior communicating arteries.

In a recent meta-analysis comprising 5100 patients conducted by Angeloni et al. [63, 64] twenty-eight studies were analyzed with a total of 1894 patients receiving unilateral ACP versus 3206 receiving bilateral ACP. Pooled analysis showed similar rates of 30-day mortality (8.6% versus 9.2% for unilateral ACP and bilateral ACP, resp.; *p* = 0.78), PND (6.1% versus 6.5%; *p* = 0.80), and TND (7.1% versus 8.8%; *p* = 0.46).

Previous studies comparing unilateral with bilateral antegrade perfusion [65–67] are discordant and ineffectual to reach a final conclusion [64]. The first study published in 2006 [66] involved only 65 patients. The stunning differences in mortality rates between bilateral ACP (12%) and unilateral ACP (1%) that could only be reached without propensity score matching were soon put into perspective if correct statistical measure was applied. The second study [67] (*n* = 280) found only an improved quality of life in patients with bilateral ACP but not significantly lower rates of mortality and/or neurologic complications.

The last report of the German Registry for Acute Aortic Dissection Type A [65] published in Circulation and including 1081 patients showed equivalent outcomes for bilateral ACP versus unilateral ACP. In accordance with this latest and largest comparative study, there is no difference in performing cerebral protection with bilateral ACP or unilateral ACP.

Those results could be supported by Vienna group of Wiedemann et al. [20]. They found no difference in the 30-day mortality (*p* = 0.59) and PND incidence (*p* = 0.699). The circulatory arrest time was slightly longer for the bilateral ACP group (29 minutes, range: 11–74 versus 33 minutes, range: 15–113; *p* = 0.023). Kaplan-Meier analysis revealed no significant differences in long-term survival between the bilateral ACP and unilateral ACP groups (1-, 3-, and 5-year survival rate: 90%, 81%, and 73% versus 79%, 77%, and 77%, resp.; *p* = 0.885).

### 3.3. Moderate versus Deep Hypothermia

DHCA has been widely used with or without adjunctive cerebral perfusion and is considered by many experts to be the standard of care for surgical repair of acute aortic dissection [14, 15, 55, 68]. However, because of the potential side effects of profound hypothermia on bypass, there has been increasing interest in performing aortic arch surgery using warmer temperatures with selective antegrade cerebral perfusion [69–72]. Avoiding profound hypothermia is associated with a reduction in bypass times, postoperative bleeding, requirement for blood transfusions in the clinical setting, and a reduction in endothelial cell dysfunction and neuronal apoptosis in the experimental setting [33, 73–75]. Consequently, a growing tendency to increase the body temperature during circulatory arrest with ACP has recently been reported from various institutions [31]. Studies in animal models have convincingly shown that cerebral oxygen consumption decreases by 50% of baseline at 28°C core body temperature. Further cooling does not effectively decrease brain oxygen consumption and neuronal metabolism [76]. Moreover, profound hypothermia impairs cerebral autoregulation and vasoconstriction decreases regional cerebral blood flow in selective ACP [77].

When comparing profound versus moderate hypothermic arrest with selective ACP during acute aortic dissection repair, Algarni et al. [59] from the Toronto General Hospital found that moderate hypothermia was independently associated with a lower risk of a composite outcome of mortality and major adverse cardiac and cerebrovascular events. The composite outcome of mortality, low cardiac output syndrome, or stroke was higher in the profound hypothermia group (52.8% versus 24%, *p* < 0.001) and cardiopulmonary bypass times and blood transfusions were significantly higher (*p* = 0.04). The authors even concluded that profound hypothermia was an independent predictor of composite outcome by multivariable analysis (odds ratio: 7.6; 95% confidence interval: 3.0–21.1).

Kamiya et al. [33] in their propensity score analysis on 377 patients found no significant differences in mortality or morbidity between deep and moderate lower body circulatory arrest, in either the entire study cohort or the propensity-matched cohort. Results suggest that moderate lower body circulatory arrest can be safely performed for aortic arch repair and postoperative inflammatory responses tended to be lower in patients with moderate lower body circulatory arrest than those with deep lower body circulatory arrest. Zierer et al. [31] reported their impressive 1002-patient single-center experience in 2012 using selective ACP with mild (28–30°C) hypothermic arrest for arch replacement and stated that the use of selective ACP makes deep hypothermia nonessential for aortic arch replacement. Their results suggest that ACP/MHCA can be safely applied to complex aortic arch surgery even in a subgroup of patients with up to 90 minutes of ACP. Very recently Leshnower et al. [23] from Emory University in Atlanta found in their cohort of 288 patients who underwent axillary artery cannulation and selective unilateral antegrade perfusion in moderate hypothermic versus deep hypothermic arrest (DHCA 21.6 ± 3.1°C versus MHCA 27.4 ± 1.6°C, *p* < 0.01) no differences in cardiopulmonary bypass, cross-clamp, or HCA times. Mortality was 14.6% for DHCA patients and 9.2% for MHCA patients (*p* = 0.17). There was no significant difference in stroke, temporary neurologic dysfunction, or dialysis-dependent renal failure.

## 4. Discussion

The optimal cerebral protection strategy to prevent brain injury during complex aortic arch surgery is an area of active interest. It is generally accepted that neurologic complications are one of the most devastating complications in cardiovascular surgery [36]. The incidence of PND in patients undergoing aortic surgery is reported to be 5% [78] but is approximately twice as high in patients undergoing aortic arch surgery [11, 79, 80]. It is well known that PND is associated with longer ventilation times and prolonged intensive care unit and hospital lengths of stay [81]. Therefore, the optimal strategy to provide best possible neuroprotection even in complicated aortic pathologies and long ischemia times becomes increasingly important. One of the most challenging aspects of comparing patient cohorts with acute dissections requiring circulatory arrest is the uncertainty of the extent of aortic replacement and other concomitant procedures that are required to ensure patient survival. Often these decisions are made intraoperatively after the aortic intima has been examined from the level of the valve to the left subclavian artery. Therefore, the operations performed to repair acute dissections can be highly variable, making it difficult to create homogenous groups of patients for the purpose of comparing various perfusion strategies.

Probably the most essential question to address is which cerebral protective strategy to offer for which patient population and under which circumstances. Important variables are the extent of aortic disease (hemiarch versus total arch), the urgency of surgical intervention (dissection with malperfusion versus chronically expanding aneurysm), and the expected duration of circulatory arrest.

The Emory group recently analyzed their experience of 708 patients who had undergone aortic arch surgery since 2004 [71]. Five hundred patients had hemiarch replacement at temperatures of 22°C with unilateral ACP. Leshnower et al. [71] propensity matched 277 patients who had undergone hemiarch replacement at more moderate temperatures of 28.6°C with 233 patients who had undergone hemiarch replacement at an average temperature of 24.3°C. They found similar operative mortalities for elective and urgent cases, no difference in the incidence of temporary neurological deficits, and a similar reoperation rate for bleeding complications. However, patients with moderate versus deep temperature management had a significantly lower rate of PND (2.5 versus 7.2%; *p* = 0.01), which was confirmed by propensity score analysis (odds ratio of 0.28; *p* = 0.02). In fact, many are progressively moving towards the new perfusion strategy of ACP and more moderate perfusion temperatures. This paradigm shift is driven by the promising results advocating the routine use of moderate-to-mild (28–35°C) hypothermia during aortic arch operations. Consequently, a growing tendency to increase the body temperature during circulatory arrest with ACP has recently been reported from various institutions [31]; however, care has to be taken regarding safe ischemic limits. The temperature relationship for the safe interruption of blood flow has been considered similar for the brain and the spinal cord; however, the absolute times for safe ischemia for the brain and spinal cord differ because of a 4-fold difference in baseline metabolism at normothermia of 37°C (5 min for the brain versus 20 min for the spinal cord) [76]. This has to be considered given the fact that not only the brain has to be protected during circulatory arrest and as shown by Etz et al. [82] moderate hypothermia (28°C) clearly has safety limits with regard to spinal cord integrity. Furthermore high body core temperatures are difficult to correct during the procedure—in the case of unpredicted technical problems—and only a minority of experienced centers so far use additional distal perfusion.

In terms of prolonged circulatory arrest (>40 min) a study conducted by the Bern University Hospital in Switzerland [67] including 129 patients with unilateral and 162 patients with bilateral perfusion suggests an advantage for bilateral. Malvindi et al. [83] also concluded that bilateral ACP may be favorable in cases of prolonged circulatory arrest durations (>40–50 min) after comparing several studies on aortic arch surgery, including more than 3500 patients treated with either unilateral (*n* = 599) or bilateral (*n* = 2949) ACP.

There is evidence that bilateral ACP with hypothermic arrest is currently the best method for cerebral protection, particularly in more complex cases of total arch replacement (>30–40 min), but unilateral ACP may be adequate if circulatory arrest is limited [36]. Given the importance of neuroprotection, recent published data have called for a consensus regarding cerebral protection during aortic arch surgery, specifically pertaining to the optimal adjunctive cerebral perfusion strategy and patient temperature. A uniform terminology of the different stages of hypothermia to allow for better comparison as well as a clear definition of the extent of the procedure to be undertaken (e.g., hemiarch/total arch; moderate hypothermia/deep hypothermia) appears essential to facilitate discussion among experts in the field and helps guide future path of modern arch surgery.

When DHCA gained widespread acceptance as the standard approach for arch surgery, antegrade cerebral perfusion (ACP) as an adjunct to deep hypothermic arrest began its triumphal march offering both improved neuroprotection and operative outcomes. This encouraged the use of ACP in combination with steadily increasing core body temperatures, cumulating in the advocation of moderate-to-mild temperatures up to 35°C. The impetus for progressive temperature elevation was the limitation of adverse effects of profound hypothermia and the most welcome side effect of significantly shorter cooling and rewarming periods, potentially alleviating systemic inflammatory responses, that is, impaired coagulation. However, the safe limits of prolonged circulatory arrest have not yet been clearly defined. In light of those recent developments, trading effective neuroprotection and excellent outcomes for the risk of prolonged “warm” ischemia might constitute a “new” risk factor, jeopardizing central nervous system integrity, especially of those undergoing extensive arch repair or with previous neurologic deficits.

Despite sophisticated and increasingly individualized surgical approaches for complex aortic pathologies, there remains a lack of consensus regarding the optimal method of cerebral protection and circulatory management during the time of arch exclusion.

## Figures and Tables

**Figure 1:** Various techniques for unilateral and bilateral antegrade cerebral perfusion. (a) Schematic presentation of an isolated ascending aortic aneurysm. (b) Unilateral ACP using direct arterial cannulation of the axillary artery. (c) Bilateral ACP with perfusion of the axillary artery and the left common carotid artery with a balloon cannula. (d) Antegrade bicarotid perfusion with two balloon occlusion cannulas.

**Table 1:** Calculated safe durations of HCA at different temperatures with regard to cerebral metabolic rate and by McCullough et al. [30].

Temperature (°C)/level of hypothermia	Cerebral metabolic rate (% of baseline)	Calculated safe duration of HCA (min)
37 (normothermia)	100	5
30 (moderate)	56 (52–60)	9 (8–10)
25 (deep)	37 (33–42)	14 (12–15)
20 (profound)	24 (21–29)	21 (17–24)
15 (profound)	16 (13–20)	31 (25–38)
10 (ultra profound)	11 (8–14)	45 (36–62)

**Table 2:** Best evidence papers.

Number of patients	Perfusion strategy	Temperature (°C)	Circulatory arrest time (min), mean ± SD or median (range)	In-hospital mortality *n* (%)	PND *n* (%)	TND *n* (%)	Ref.
1002	ACP/MHCA	30.0 ± 2.0	36.0 ± 19.0	52.0 (5.0)	28.0 (3.0)	42.0 (4.0)	[31]
412		25.7 ± 2.8	30 ± 15	29 (7.0)	15 (3.6)	21 (5.1)	[32]
252		26.3 ± 0.9	23.5 ± 15.8	20.0 (7.9)	13.0 (5.1)	32.0 (12.6)	[33]
206		27.4 ± 1.6	39.0 ± 20.0	19.0 (9.2)	17.0 (8.3)		[23]
47		25.9 ± 1.6	28.0 ± 6.0	7.0 (14.9)	1.0 (2.1)	10.0 (21.3)	[34]

7038	ACP/DHCA	24.2 ± 3.2		5.9%	7.0%	3.8%	[35]
125		23.2 ± 1.2	34.1 ± 24.4	14.0 (11.2)	10.0 (8.0)	28.0 (22.4)	[33]
91			30.0 (14.0–92.0)	12 (13.0)	11 (12.0)	2 (2.0)	[20]
88		21.6 ± 2.1	37.0 ± 20.0	12.0 (14.6)	7.0 (8.5)		[23]
51		20.0 ± 2.2	31.5 ± 5.7	10.0 (19.2)	2.0 (3.8)	21.0 (40.4)	[34]

242	bACP/DHCA	25.0 ± 4.0	23.0 ± 21.0	34 (14.0)	20 (8.3)	36 (14.9)	[36]
123	uACP/DHCA	24.0 ± 3.0	22.0 ± 17.0	9 (7.3)	13 (10.6)	22 (17.9)	[36]

1141	RCP/DHCA	21.2 ± 3.7		7.2%	8.5%	4.4%	[35]
122			30.0 (14.0–88.0)	20 (16.0)	15 (12.0)	0 (—)	[20]
51		23.0 ± 3.0	18.0 ± 12.0	4 (7.8)	8 (15.7)	9 (17.6)	[36]

220	DHCA	22.0 ± 2.0	15.0 ± 13.0	25 (11.4)	31 (14.1)	28 (12.7)	[36]
116			36.0 (12.0–88.0)	30 (26.0)	27 (23.0)	1 (1.0)	[20]
